# Decision-Making for the Lifetime Performance Index

**DOI:** 10.1155/2021/3005067

**Published:** 2021-07-12

**Authors:** Basim S. O. Alsaedi, M. M. Abd El-Raouf, E. H. Hafez, Zahra Almaspoor, Osama Abdulaziz Alamri, Kamel Atallah Alanazi, Saima Khan Khosa

**Affiliations:** ^1^Department of Statistics, Faculty of Science, University of Tabuk, Tabuk, Saudi Arabia; ^2^Basic and Applied Science Institute, Arab Academy for Science, Technology and Maritime Transport (AASTMT), Alexandia, Egypt; ^3^Department of Mathematics, Faculty of Science, Helwan University, Cairo, Egypt; ^4^Department of Statistics, Yazd University, P. O. Box 89175-741, Yazd, Iran; ^5^University of Jeddah, Faculty of Science and Arts (Al Kamil), Department of Mathematics, Jeddah, Saudi Arabia; ^6^Department of Statistics, Bahauddin Zakariya University, Multan, Pakistan

## Abstract

The purpose of this research is to develop a maximum likelihood estimator (MLE) for lifetime performance index *C*_*L*_ for the parameter of mixture Rayleigh-Half Normal distribution (RHN) under progressively type-II right-censored samples under the constraint of knowing the lower specification limit (*L*). Additionally, we suggest an asymptotic normal distribution for the MLE for *C*_*L*_ in order to construct a mechanism for evaluating products' lifespan efficiency. We have specified all the steps to carry out the test. Additionally, not only does hypothesis testing successfully assess the lifetime performance of items, but it also functions as a supplier selection criterion for the consumer. Finally, we have added two real data examples as illustration examples. These two applications are provided to demonstrate how the results can be applied.

## 1. Introduction

Process capability analysis is an efficient method for determining a production process's performance and prospective capabilities. In manufacturing sectors, process capability indices (PCIs) are used to determine if the quality of the product meets specified standards. PCIs have garnered considerable interest in the statistical literature during the last three decades. The key motivation for analyzing the process capacity producing PCI is to evaluate the process's performance and potential capabilities.

Process capability analysis aids in the following ways: continuously monitoring process quality using PCI to ensure produced goods adhere to requirements, giving information on product development to manufacturers and specialists, and establishing a foundation for lowering item failures. The PCIs are classified into three categories: the first is used to quantify the target-the-better quality feature, the second is used to quantify the larger-the-better quality characteristic, and the third is used to quantify the smaller-the-better quality characteristic. For more information and extra details, see [1].

Due to a variety of variables such as time limits or other constraints on money, material resources, or data collection, the researcher may be unable to track the lifespan of all commodities or things in a test. As a result, it is possible that censored samples will be encountered during operation. Proper filtering happens when just the lifetime's lower limit is known. When only the lifetime cutoff is set, proper filtering occurs. One type of right censorship is referred to as “type-II censorship.” This type of censorship may occur when a certain number of failures occur during the lifespan experiment.

Progressive type-II censorship occurred when our attention shifted from monitoring *n* goods to monitoring until the *m*^th^ failure occurs, and then, the test is ended. As the *i*^th^ item fails, *r*_*i*_ of the items that still functional are cut off from the experiment. At the end of the experiment, the lasting *r*_*m*_=*n* − *m* − ∑_*i*=1_^*m*^*r*_*i*_ are eliminated at the time of the *m*^th^ item which is failed. For more information and extensive reading, see [2] and [3]. For more reading, see [4–8].

Typically, a high sample size is required in practice to evaluate the product's effectiveness under nonnormal distributions, and this study used a large sample size and an increasing proportion of type-II right-censored samples. Using a large sample size and an increasing proportion of type-II right-censored samples, this study created a novel method for assessing a product's performance improvement when the distribution is nonnormal.

Thus, the primary objective of this work is to estimate *C*_*L*_'s MLE under the parameter RHN distribution using a type-II right-censored sample.

A confidence interval is then constructed using the asymptotic normal distribution of the MLE of *C*_*L*_. Additionally, we use confidence intervals to construct a unique hypothesis testing approach for evaluating items' lifetime performance. The novel hypothesis testing approach may be used to evaluate the quality performance of items with nonnormal distribution using large sample size and an increased role of type-II right-censored items. Additionally, purchasers may employ the unique hypothesis testing procedure to determine whether the manufacturer's lifetime falls within the defined range. Additionally, vendors can leverage the unique hypothesis testing approach to enhance the capability of their processes.

## 2. Finite Mixture of Rayleigh and Half-Normal Distribution

Pearson [9] is credited with inventing statistical modelling using finite mixtures of distributions when he applied the concept to a study of crab morphometry data provided by Weldon [10, 11]. The dataset consisted of 1000 cm of measurements of the ratio of the forehead to the body length. The data were skewed to the right when plotted. Weldon [11] claimed that this skewness might be explained by the fact that the sample includes members of two distinct crab species, but no such distinction had been noted at the time the information was gathered. Pearson [9] proposed that a weighted sum of two normal distributions may be used to simulate the distribution of data, with the two weights representing the percentage of each variety of crab.

The Rayleigh-Half Normal distribution is denoted as RHN(*θ*) by Abd El-Monsef and Abd El-Raouf [12]. This model is a combination of Rayleigh and Half-Normal distributions, each with different parameters $\left(1/\sqrt{2\theta }\right)$, where *f*_*R*_ refers to the pdf of the Rayleigh distribution and *f*_HN_ refers to the pdf of Half-Normal distribution:

(1) $$\begin{array}{c} f\left(x,\theta \right)=Kf_{R}\left(\frac{x\cdot 1}{\sqrt{2\theta }}\right)+\left(1-K\right)f_{\text{HN}}\;\left(\frac{x\cdot 1}{\sqrt{2\theta }}\right)\\ =K\left(2\theta xe^{-\theta x^{2}}\right)+\left(1-K\right)\left(2\;\sqrt{\frac{\theta }{\pi }}\;e^{-\theta x^{2}}\right), \end{array}$$

where $K=\left(1/\left(1+\sqrt{\pi \theta }\right)\right)$.

A Rayleigh-Half Normal distribution has a pdf that looks like the following:

(2) $$\begin{array}{c} f\left(x,\;\theta \right)=\frac{2\theta \left(x+1\right){\text{e}}^{-\theta x^{2}}}{1+\sqrt{\pi \theta }},\;x\cdot \theta >0. \end{array}$$

### 2.1. The LPI of RHN Distribution

The electronic components' lifespan performance is evaluated using the *C*_*L*_ process capability index, which was introduced by [13]. Better quality indicates a longer lifespan. Typically, lifespan requirements must be met with at least *L* units of lifespan. In order to judge the product efficiency, the lifespan performance index *C*_*L*_ is described this way:

(3) $$\begin{array}{c} C_{L}=\frac{\mu -L}{\sigma }, \end{array}$$

where $\mu =\left(2\sqrt{\theta }+\sqrt{\pi }\right)/\left(2\sqrt{\theta }\left(1+\sqrt{\pi \theta }\right)\right)$ denotes the mean of RHN distribution, $\sigma =\sqrt{\left(\left(4-\pi +2\sqrt{\pi \theta }+2\theta \left(\pi -2\right)\right)/4\theta {\left(1+\sqrt{\pi \theta }\right)}^{2}\right)}$ represents the standard deviation of RHN distribution, and *L* denotes the well-defined lower specification limit. A case may be made that the lifetime of items can be represented using the RHN distribution. The performance index used for determining product performance is specified as *C*_*L*_. If *X* originates with (RHN) distribution, *C*_*L*_ is an index that accounts for a lifetime of superior performance:

(4) $$\begin{array}{c} C_{L}=\frac{\sqrt{\pi }+2\sqrt{\theta }-2L\left(\sqrt{\theta }-\sqrt{\pi }\theta \right)}{\left(\sqrt{\theta }+\sqrt{\pi }\theta \right)\sqrt{\left(4\left(1-\theta \right)+2\sqrt{\pi \theta }+\pi \left(2\theta -1\right)\right)/\theta {\left(1+\sqrt{\pi \theta }\right)}^{2}}};\;\theta >0, \end{array}$$

where −*∞* < *C*_*L*_ < (*μ*/*σ*).

As can be seen, the mean is inversely related to the rate of failure and directly related to the greater *C*_*L*_ > 0, which is LPI. As a result, *C*_*L*_ provides an accurate representation of the lifetime development of existing new products.

## 3. The Conforming Rate for RHN Distribution

Suppose that if the lifespan of an item or units under testing is *X* and the lower bound is *L*, so we can say that the item is regarded to be compliant, when its lifetime exceeds *L*. The complying rate expresses the likelihood of conforming goods and may be defined as

(5) $$\begin{array}{c} P_{r}=P\left(x\geq L\right). \end{array}$$

From equation (3), *L*= *μ* − *σ* *C*_*L*_, and by substituting in (5), we obtain

(6) $$\begin{array}{c} P_{r}=1+\left(\frac{e^{-\left(\theta M^{2}/4\right)}-\sqrt{\pi \theta }\text{ erf}\left(\sqrt{\theta }M/2\right)-1}{1+\sqrt{\pi \theta }}\right), \end{array}$$

where

(7) $$\begin{array}{c} M=\left(\frac{1}{\theta }\;C_{L}\sqrt{\frac{4\left(1-\theta \right)+2\sqrt{\pi \theta }+\pi \left(2\theta -1\right)}{\theta {\left(1+\sqrt{\pi \theta }\right)}^{2}}}\frac{2\theta -1}{\theta +\sqrt{\pi }\theta^{3/2}}\right). \end{array}$$

Using the one-to-one link between *P*_*r*_ and *C*_*L*_, the index of lifetime performance can be a versatile and effective tool for evaluating the product's quality as well as estimating the complying rate *P*_*r*_. *P*_*r*_ versus *C*_*L*_ is determined for various values of parameters, as shown in Tables 1 and 2.

Obviously, the complying rate *P*_*r*_ and the *C*_*L*_ can exhibit a strictly rising connection. Tables 1 and 2 show different *C*_*L*_ values and their corresponding complying rates *P*_*r*_ for parameters of *θ* equal to 0.5 and 1.768.

## 4. The MLE for *C*_*L*_

Let us assume that we have a random sample for our distribution ordered and it is organized as follows:*X*_1:*m*:*n*:*k*_, *X*_2:*m*:*n*:*k*_,…, *X*_*m*:*m*:*n*:*k*_. This sample represents the appropriate progressive type-II right-censored sample from a real practical experiment for *n* units with survival times distributed according to the RHN distribution, and *r*=(*r*_1_, *r*_2_,…, *r*_*m*_) represents the censoring scheme that items under experiment will be removed according to it. Then, the likelihood function of all *m* progressively type-II right-censored order statistics is expressed as follows:

(8) $$\begin{array}{c} L\left(x,\theta \right)=Ck^{m}\prod_{i=1}^{m}f_{X}\left(x_{i:m:n:k};\;\theta \right){\left(1-F_{X}\left(x_{i:m:n:k};\;\theta \right)\right)}^{k\left(r_{i}+1\right)-1}, \end{array}$$

where 0 < *x*_1:*m*:*n*:*k*_ <  *x*_2:*m*:*n*:*k*_ < ⋯<*x*_*m*:*m*:*n*:*k*_ < *∞* and *C*=*n*(*n* − *r*_1_ − 1)(*n* − *r*_2_ − 1) ⋯ (*n* − ∑_*i*=1_^*m*−1^*r*_*i*_ − *m*+1).

Now, we will get the MLE for the RHN distribution parameters, by finding the first derivative for the likelihood function as follows:

(9) $$\begin{array}{c} \frac{\partial l\left(x,\theta \right)}{\partial \theta }=\frac{m}{\theta }-\frac{m\sqrt{\pi }}{2\sqrt{\theta }Q}-\overset{m}{\underset{i=1}{\sum }}x_{i}^{2}+\overset{m}{\underset{i=1}{\sum }}\frac{\left(k\left(1+r_{i}\right)-1\right)\left(\left(\sqrt{\pi }S/2\sqrt{\theta }Q\right)-W\right)}{Q-S}=0, \end{array}$$

where $S=\left(1-e^{-\theta x_{i}^{2}}+\sqrt{\pi \theta }\text{erf}\left(\sqrt{\theta }x_{i}\right)\right)$,

(10) $$\begin{array}{c} W=\frac{\sqrt{\pi }\text{erf}\left(\sqrt{\theta }x_{i}\right)}{2\sqrt{\theta }}+x_{i}e^{-\theta x_{i}^{2}}+x_{i}^{2}e^{-\theta x_{i}^{2}}, \end{array}$$

and $Q=1+\sqrt{\pi \theta }$ and the MLE $\hat{\theta }$ of *θ* can be obtained numerically.

By the aid of the invariance property of MLE that was introduced by Zehna [14], we can obtain the MLE of *C*_*L*_ as shown below:

(11) $$\begin{array}{c} {\hat{C}}_{L}=\frac{\sqrt{\pi }+2\sqrt{\hat{\theta }}-2L\left(\sqrt{\hat{\theta }}-\sqrt{\pi }\hat{\theta }\right)}{\left(\sqrt{\hat{\theta }}+\sqrt{\pi }\hat{\theta }\right)\sqrt{\left(\left(4\left(1-\hat{\theta }\right)+2\sqrt{\pi \hat{\theta }}+\pi \left(2\hat{\theta }-1\right)\right)/\hat{\theta }{\left(1+\sqrt{\pi \hat{\theta }}\right)}^{2}\right)}}. \end{array}$$

Furthermore, the asymptotic normal distribution for MLEs is stated and published by Soliman [15] and Wu and Kuş [3].

As a first step, we get the observed Fisher information of the parameter *θ*:

(12) $$\begin{array}{c} I\left(\hat{\theta }\right)=-\frac{m\left(4+7\sqrt{\pi \theta }+2\pi \theta \right)\left(-1+k+kr_{i}\right)}{4{\left(\theta +\sqrt{\pi }\theta^{3/2}\right)}^{2}}\\ {}*\overset{m}{\underset{i=1}{\sum }}\left(-\frac{{\left(-\left(W/Q\right)+\left(\sqrt{\pi }S/2Q^{2}\sqrt{\theta }\right)\right)}^{2}}{{\left(1-\left(S/Q\right)\right)}^{2}}+\frac{-\left(\sqrt{\pi }S/4Q^{2}\theta^{3/2}\right)-\left(\pi S/2Q^{3}\theta \right)+\left(\sqrt{\pi }W/Q^{2}\sqrt{\theta }\right)-\left(\left(-\left(\sqrt{\pi }\text{erf}\left(\sqrt{\theta }x_{i}\right)/4\theta^{3/2}\right)+\left(x_{i}e^{-\theta x_{i}^{2}}/2\theta \right)-x_{i}^{3}e^{-\theta x_{i}^{2}}-x_{i}^{4}e^{-\theta x_{i}^{2}}\right)/Q\right)}{1-\left(S/Q\right)}\right). \end{array}$$

The asymptotic distribution of MLE $\hat{\theta }$ is a normal distribution with mean *θ* and the asymptotic variance $I^{-1}\left(\hat{\theta }\right)$ is denoted by $N\left(\theta ,I^{-1}\left(\hat{\theta }\right)\right)$. So, the lower and upper bounds for the distribution parameter *θ* is denoted by $\hat{\theta }\pm z_{\alpha /2}\sqrt{I^{-1}\left(\hat{\theta }\right)}$.

Depending on the Delta method [16], we can get that the asymptotic distribution for *C*_*L*_ ≡ *h*(*θ*) is the asymptotic normal distribution of $h\left(\hat{\theta }\right)$ with mean *C*_*L*_ and asymptotic variance Σ_*θ*_ as

(13) $$\begin{array}{c} {\hat{C}}_{L}\equiv h\left(\hat{\theta }\right)∼N\left(C_{L},\Sigma_{\theta }\right), \end{array}$$

where $\Sigma_{\theta }=I^{-1}\left(\theta \right){\left[\partial h\left(\theta \right)/\partial \theta \right]}_{\theta =\hat{\theta }}^{2}$.

## 5. Step Followed and Procedure for Obtaining *C*_*L*_

The statistical analysis hypothesis testing approach is used to determine if the LPI is within the specified range. By incorporating Lee et al. [17–19], the confidence interval and hypothesis testing may be obtained, for more extra reading we can refer to Lee et al. [17–21].

We can obtain *C*_*L*_ confidence interval by considering ${\hat{C}}_{L}$ distributed normally having mean *C*_*L*_ and asymptotic variance (Σ_*θ*_). Assuming that the needed value of the LPI is greater than *c*^*∗*^, where *c*^*∗*^ signifies the intended value, the null hypothesis is tested as follows.

 
*H*_*o*_ :  *C*_*L*_ ≤ *c*^*∗*^ against *H*_1 _ :  *C*_*L*_ > *c*^*∗*^.

Due to the fact that the MLE of *C*_*L*_ is utilised as the test statistic, the rejection area may be calculated as follows: $\left[{\hat{C}}_{L}>\left(C_{0}/C_{L}\right)\right]$. For a given significance level *α*, the critical value *C*_0_ is calculated as follows:

(14) $$\begin{array}{c} P\left({\hat{C}}_{L}>\frac{C_{0}}{C_{L}}=c^{*}\right)=\alpha ,\\ P\left({\hat{C}}_{L}-C_{L}\leq \frac{C_{0}-C_{L}}{C_{L}}=c^{*}\right)=1-\alpha ,\\ P\left(\frac{{\hat{C}}_{L}-C_{L}}{\sqrt{\Sigma_{\hat{\theta }}}}\leq \frac{C_{O}-c^{*}}{\sqrt{\Sigma_{\hat{\theta }}}}\right)=1-\alpha ,\\ P\left(\frac{{\hat{C}}_{L}-C_{L}}{\sqrt{\hat{\Sigma_{\theta }}\;}}\leq \frac{C_{O}-c^{*}}{\sqrt{\hat{\Sigma_{\theta }}\;}}\right)=1-\alpha , \end{array}$$

where $\left(\left(\hat{C_{L}}-C_{L}\right)/\sqrt{\hat{\Sigma_{\theta }}\;}\right)∼N\left(0,1\right)$.

Such that **z**_*α*_ is the standard normal value, so we can express it as $z_{\alpha }=\left(\left(C_{O}-c^{*}\right)/\sqrt{\hat{\Sigma_{\theta }}\;}\right)$, so the critical value may be expressed as follows:

(15) $$\begin{array}{c} C_{O}=c^{*}+z_{\alpha }\sqrt{\hat{\Sigma_{\theta }}\;}, \end{array}$$

where *c*^*∗*^, *α*, and $\hat{\Sigma_{\theta }}$ denote the target value. Additionally, we discover that *C*_*O*_ is independent of *n* and *r*_*i*_,  *i*=1; 2; …, *m*. Moreover, the 100(1 − *α*)% confidence interval of *C*_*L*_ may be expressed as follows:

(16) $$\begin{array}{c} C_{L}\geq {\hat{C}}_{L}-z_{\alpha }\sqrt{\hat{\Sigma_{\theta }}}. \end{array}$$

And, *C*_*L*_ lower bound may be expressed as follows:

(17) $$\begin{array}{c} \underline{\text{LB}}=\;{\hat{C}}_{L}-z_{\alpha }\sqrt{\hat{\Sigma_{\theta }}}. \end{array}$$

The managers may use the unilateral confidence interval to detect if product performance reaches the desired level.

The testing approach for *C*_*L*_ is as follows:

  The MLE of the RHN distribution's parameters is quantitatively determined.
  Determine the lowest lifespan *L* for goods and the lifetime *c*^*∗*^ index.
  After that we construct the null and the alternative hypothesis as shown *H*_*o*_ : *C*_*L*_ ≤  *c*^*∗*^*H*_1 _ : *C*_*L*_ >  *c*^*∗*^ is constructed. By taking into consideration, a certain prespecified value of (*α*).
  Specify the number of observed failures before the test reaches an end, let us say *m*, and specify the number of the censored units according to the censoring scheme *r*= (*r*_1_, *r*_2_,…, *r*_*m*_).
  After that, we calculate the lower bound *L*.
  The statistical test decision rule may be established as if the lifetime index value *c*^*∗*^ ∉ [LB,*∞*), so we must not accept *H*_*o*_.

An indicator is given of the product lifespan index at the desired level. The quality performance of nonnormal distribution products with a big sample and more type-II right-censored samples may also be evaluated as per the hypothesis test process. Moreover, not only can the product lifetime performance be assessed appropriately but also the hypothesis test technique is the criterion for customer choice by the provider.

## 6. Numerical Examples

Hypothesis testing methodologies may be used to assess whether a product's lifetime performance remains within the specified range. A procedure is proposed in the presented study of the test, which is based on a one-sided confidence interval under RHN distribution and increasingly type-II right-censored sample. The following two examples will be applied to demonstrate the use of these hypothesis testing procedures.

**Example 1 .**

The statistics on the failure times of 24 ball bearings in an endurance test are presented, the simulated data are produced from the RHN distribution with *c*=6, *k*=4, *n*=24,  and *m*=10, and the specified censoring scheme *r*={0,0,0,1,0,0,0,0,1,3}. The observations are *x*_*i*:10:24_, *i*=1,2,…, 10=0.0002,  0.0003,  0.0006,  0.0007,  0.0063,  0.0131,  0.0303,  0.0566,  0.2669,  0.2840, respectively.

A type-II right-censored sample was considered on size of sample *m*=10 from the original set of data of 24 observations of ball bearings in a survival test.

Then, the suggested testing technique for *C*_*L*_ can be carried out as follows:

By considering the increasingly type-II right-censored sample (*x*_*i*:10:24_;  *i*=1,2,…, 10) and (*r*_1_, *r*_2_,…, *r*_10_), the MLE $\hat{\theta }$ of *θ* can be attained numerically, $\hat{\theta }=0.23696$.
If the lower lifetime limit *L* is set to 0.005, the item bearing is considered to be a conforming product.
To address product-related problems about operational performance and conformance rate *P*_*r*_ of goods must be more than 80 percent, the *C*_*L*_ value is mandatory to exceed 0.8. Thus, the value of LPI is set at *c*^*∗*^= 0.9168.
The testing hypothesis: *H*_*o*_ : *C*_*L*_ ≤ 0.9168 vs. *H*_1 _ : *C*_*L*_ >  0.9168 is constructed with specifying a significance level *α* = 0.05.
The asymptotic variance $\hat{\Sigma_{\theta }}$ and the lifetime performance estimates ${\hat{C}}_{L}$ are obtained $\hat{\Sigma_{\theta }}=0.000926795\text{ and }{\hat{C}}_{L}=1.54825$.
Then, 95% of the lower confidence interval bound can be calculated as
  (18) $$\begin{array}{c} \underline{\text{LB}}=1.54825-1.645\sqrt{0.000926795}=1.49817. \end{array}$$
So, we can easily obtain the 95% confidence interval for ${\hat{C}}_{L}$, which is $\left[\underline{\text{LB}},\infty \right)\left(=\left[1.49817,\infty \right)\right)$.
In addition, we calculate ${\hat{C}}_{L}=1.54825>C_{O}=c^{*}+z_{\alpha }\sqrt{\hat{\Sigma_{\theta }}\;}=0.9168+1.645\sqrt{0.000926795}=0.9669$, so we also reject *H*_*o*_ : *C*_*L*_ ≤ 0.9168.

From the obtained results, it can be noticed that the value of the performance index $c^{*}=0.9168\notin \left[\underline{\text{LB}},\infty \right)$; thus, *H*_*o*_ : *C*_*L*_ ≤  0.9168 is rejected. Hence, there is a suggestion to indicate that the LPI of 24 items' bearing operation does meet the mandatory level.

**Example 2 .**

The simulated data is an increasingly type-II censored sample from the RHN distribution. The 30 experimental units are located simultaneously in a lifetime test with *c*=6, *k*=2, *n*=30, *m*=20 and the given censoring scheme is *r*={ 0,  0,  0,  2,  0,  0,  0,  2,  0,  0,  0,  2,  2,  0,  0,  0,  0,  0,  0,  2}. The progressively type-II censored sample is *x*= {0.1816,  0.1958,  0.2185,  0.2516,  0.2604,  0.3074,  0.3277,  0.3381,  0.3487,  0.3595,  0.3705,  0.4165,  0.4528,  0.4779,  0.5432,  0.5702,  0.611,  0.6255,  0.7103,  0.7245}.

Then, the suggested testing technique for *C*_*L*_ can be written as follows.
Assume that we have a type-II right-censored sample *x*_*i*:20:30_,  *i*=1,2,…, 20, and (*r*_1_, *r*_2_,…, *r*_20_). The MLE $\hat{\theta }$ of *θ* can be obtained numerically, $\hat{\theta }=0.71088$.
The lower lifetime limit *L* is assumed to be 0.005.
To handle the product purchasers' concerns concerning operational performance, the conforming rate *P*_*r*_ of products is required to exceed 80 percent; the *C*_*L*_ value is required to exceed 0.82. Thus, the performance index value is set at *c*^*∗*^= 0.82.
The testing hypothesis: *H*_*o*_ : *C*_*L*_ ≤  0.82 vs. *H*_1 _ : *C*_*L*_ >  0.82 is created.
The lifetime performance estimate ${\hat{C}}_{L}$ and the asymptotic variance $\hat{\Sigma_{\theta }}$ are obtained:
  (19) $$\begin{array}{c} {\hat{C}}_{L}=1.4352,\\ \hat{\Sigma_{\theta }}=0.0007153. \end{array}$$
Then, 95% of the lower confidence interval bound can be calculated as
  (20) $$\begin{array}{c} \underline{\text{LB}}=1.4352-1.645\sqrt{0.0007153\;}=1.3912. \end{array}$$
So, we can evaluate the lower and upper bounds for the confidence interval.
In addition, we calculate ${\hat{C}}_{L}=1.4352>C_{O}=c^{*}+z_{\alpha }\sqrt{\hat{\Sigma_{\theta }}\;}=0.82+1.645\sqrt{0.0007153}=0.86399$, so we also reject *H*_*o*_ : *C*_*L*_ ≤  0.82.

As a result of the obtained results, it is clear that the performance index value $c^{*}=0.82\notin \left[\underline{\text{LB}},\infty \right)$; thus, *H*_*o*_ : *C*_*L*_ ≤ 0.82 is rejected.

## 7. Conclusions

Process capability indices are used throughout the production process to determine whether the product meets specified quality criteria. For quality characteristics where greater is preferable, the LPI *C*_*L*_ is one of the most often used capacity indices. Montgomery [10] was the first to work on this subject. The normalcy assumption is extremely problematic in the majority of processes, such as business and manufacturing despite the fact that it is commonly used in process capability analysis. As a result, it is common to see censored samples in operation. This study dedicated to assessing the LPI *C*_*L*_ of items follows the RHN distribution under right censoring data. The MLE of *C*_*L*_ was determined under the RHN distribution with the progressively type-II right-censored sample. The MLE of *C*_*L*_ was used to develop a confidence interval of *C*_*L*_ under the condition of known *L*, and the hypothesis testing procedure was performed.

Additionally, the offered study includes tables summarizing the LPI and its associated compliance rate. Thus, for any specified complying rate, a matching *C*_*L*_ must be evaluated, and the hypotheses underlying the testing technique may also be quantified in terms of complying rate if *L* is known to be a limit. The suggested approach is shown using real data, and the findings suggest that the objective of assessing the LPI was met.

## Figures and Tables

**Table 1:** Numerical values for the index of *C*_*L*_ vs. *P*_*r*_ for RHN distribution with the parameter value (*θ* = 0.5).

*C*_*L*_	*P*_*r*_
−*∞*	0.00000
−5	0.00005
−4	0.00068
−2	0.04019
−1.5	0.08550
−1	0.16397
−0.8	0.20675
−0.5	0.2857
−0.4	0.31323
−0.2	0.37652
−0.1	0.41042
0	0.44566
0.1	0.4821
0.2	0.51955
0.3	0.55785
0.4	0.59676
0.5	0.63609
0.6	0.67559
0.7	0.71503
0.8	0.75416
0.85	0.77353
0.9	0.79273
0.9168	0.81
0.95	0.81173
1	0.83051
1.1	0.86725
1.2	0.90274
1.4	0.9592
1.3	0.93676
1.5	0.99967

**Table 2:** Numerical values for the index of *C*_*L*_ vs. *P*_*r*_ for RHN distribution with the parameter value (*θ* = 1.768).

*C*_*L*_	*P*_*r*_
−*∞*	0.00000
−5	0.00008
−4	0.0012
−2	0.0135
−1.5	0.0294
−1	0.0364
−0.8	0.0408
−0.5	0.0464
−0.4	0.0568
−0.2	0.1454
−0.1	0.2525
0	0.3695
0.1	0.4069
0.2	0.4892
0.3	0.5251
0.4	0.5471
0.5	0.6123
0.6	0.6944
0.7	0.7376
0.8	0.7954
0.82	0.8017
0.85	0.8094
0.9	0.8237
0.95	0.8379
1	0.8539
1.1	0.7854
1.2	0.8846
1.4	0.9233
1.3	0.9592
1.5	0.9696

## Data Availability

All data are available within the paper.
